# Application of Medical-Nursing Integration Multidisciplinary-Assisted Surgical Wound Nursing Mode in Improving the Quality of Wound Treatment

**DOI:** 10.1155/2022/9299529

**Published:** 2022-08-30

**Authors:** Jinyan Wang, Ting Yuan, Jun Shi

**Affiliations:** ^1^Department of Obstetrics, People's Hospital of Dongxihu, District, Wuhan 430040, Hubei, China; ^2^Department of Endoscopy Center, People's Hospital of Dongxihu, District, Wuhan 430040, Hubei, China; ^3^Department of Orthopaedics, People's Hospital of Dongxihu, District, Wuhan 430040, Hubei, China

## Abstract

Surgical treatment is a common clinical intervention for trauma, but postoperative pain and poor nursing lead to slow wound recovery and wound infection. Therefore, it is extremely important to select effective nursing intervention methods to improve the quality of wound treatment. This study explored the application value of the wound care model of medical integration and multidisciplinary-assisted surgery in improving the quality of wound treatment. The results show that medical-nursing integration in multidisciplinary-assisted surgical wound nursing mode can improve the quality of wound treatment and pain level in patients, which is beneficial to improving team cohesion of medical staff and satisfaction evaluation of patients.

## 1. Introduction

Trauma is a common type of disease in general surgery. It refers to severe trauma to the body, resulting in massive hemorrhage and tissue destruction. Human tissue or organ damage is often caused by mechanical factors. In recent years, with the development of industry, agriculture, and transportation, the trauma caused by various accidents is increasing day by day [1, 2]. Surgical treatment is a common clinical intervention. Debridement, suture, and other methods can effectively promote wound healing at the local injury site. However, in some patients, postoperative pain and poor nursing lead to slow wound recovery and even cause wound infection in severe cases, which increases the difficulty of clinical treatment and medical expenses of patients [3, 4]. Therefore, it is extremely important to choose effective nursing intervention methods to improve the quality of wound management. The medical-nursing integration multidisciplinary-assisted surgical wound care model integrates medical and nursing resources and refers to a multidisciplinary cooperation model between doctors and nurses through information exchange, cooperation, and complement [5]. In this nursing model, through formulating effective nursing intervention countermeasures, the limitation of differential diagnosis and treatment can be effectively avoided, and the situation that patients travel to multiple specialist outpatient clinics after injury can be avoided, thus realizing meticulous management of wound recovery. At present, this nursing model has achieved good nursing results in ophthalmology and oncology, but it is rarely reported in general surgery wound care [6, 7]. Therefore, the purpose of this study was to explore the application of the medical-nursing integrated multidisciplinary-assisted surgical wound care model in improving the quality of wound treatment.

## 2. Materials and Methods

### 2.1. General Information

A total of 200 patients admitted to the general surgery department of our hospital from January 2020 to January 2022 were selected as the research subjects. 96 patients admitted from January 2020 to May 2021 were included in the control group, and 104 patients admitted from June 2021 to January 2022 were included in the observation group. There was no significant difference in baseline data between the two groups (*P* > 0.05), and they were comparable.

### 2.2. Inclusion Criteria

The inclusion criteria were as follows: age ≥18 years old and all are surgical site wounds.

### 2.3. Exclusion Criteria

The exclusion criteria were as follows: complicated with severe hepatic and renal insufficiency, critically ill with obvious signs of shock, complicated with severe infection, and incomplete clinical data.

### 2.4. Nursing Methods

The control group received routine care. After entering the department, conduct education about disease and surgery-related knowledge. During postoperative dressing change, the wounds were washed with normal saline and routinely disinfected with iodophor. Postoperative pain relief and psychological care were given, and changes in the patient's condition were monitored. After the condition was stable, routine functional exercises were guided.

Based on the control group, the observation group was combined with the medical-nursing integrated multidisciplinary-assisted surgical wound care model. (1) Establish a medical-nursing integrated multidisciplinary team to assist in surgical wound care. The head nurse is the team leader, the deputy head nurse is the deputy team leader, and a team is formed with the attending doctor, nutritionist, rehabilitation specialist, and nurses. Each member cooperates with each other and has clear responsibilities. Under the coordination of the nursing department, the pain department, nutrition department, and wound treatment specialists were organized to train the team members. The training content includes anatomical characteristics of the skin, wound types, wound healing, wound assessment, wound measurement, nutritional supplementation, pain management, and dressing selection. The training is carried out in the form of classroom lectures, group discussions, clinical practice, and case studies, to improve the theoretical and operational knowledge level of the team members. (2) Specific implementation plans: after discussion among the team members, a standardized work responsibility table, wound assessment scale, debridement, and informed consent form for special consumables were developed. After the patient is admitted to the hospital, the tube bed doctor initially assesses the wound and is responsible for surgery or arranging a referral. Surgical debridement, wound suture, and skin grafting were used for emergency treatment, and bacterial culture specimens were taken for examination. The dietitian evaluates the patient's postoperative recovery to formulate a dynamic nutritional plan and ensures the intake of nutrients through diet, intravenous, and other means. The responsible nurse nurses dynamically evaluate and use wet healing techniques (different types of dressings) for nursing and take pictures after each nursing to record the wound recovery. When the granulation tissue grows well or reaches the indications for skin grafting, discuss with the doctor and arrange two subskin grafts and sutures. According to the recovery of the patient after the operation, a personalized exercise method is developed under the guidance of a rehabilitation specialist. (3) Condition observation and feedback: the patient's general condition, including wound recovery and nutritional status, is assessed during the morning shift and ward rounds every morning, and the wound condition, including wound area, depth, and pain level of the patient, is checked together. (4) Discharge follow-up: for patients who have reached the indication for discharge but the wound has not yet healed, continue to follow-up and observe, conduct follow-up by telephone or WeChat once a week, understand the recovery of the patient's wound through subjective descriptions and pictures, and provide daily self-care if necessary, which includes rehabilitation training instruction, diet instruction, wound nursing method instruction, and psychological nursing. Both groups continued nursing for two weeks.

### 2.5. Observation Indicators

#### 2.5.1. Comparison of Wound Repair Levels between the Two Groups of Patients

The wound repair conditions, including wound area, wound depth, and pain level, were compared between the two groups before surgery, after 2 weeks of nursing, and after 4 weeks of nursing. The pain was evaluated using visual analog scoring (VAS), which was scored by a walking scale about 10 cm in length, with 0 indicating no pain and 10 indicating the most severe pain that was unbearable [8].

#### 2.5.2. Comparison of Wound Healing between Two Groups of Patients

The time of granulation growth, the number of dressing changes, and the time of wound healing were compared between the two groups.

#### 2.5.3. Comparison of the Incidence of Complications between the Two Groups of Patients

The incidence of complications during treatment, including wound exudation, wound bleeding, nerve damage, and joint stiffness, were compared between the two groups.

#### 2.5.4. Comparison of Patient Satisfaction Evaluation between Two Groups

When the patient was discharged from the hospital, the self-made satisfaction evaluation questionnaire was used to evaluate the patient's satisfaction, including four items of the hospital environment, medical and nursing professional level, work attitude, and psychological care. Each item was 100 points. A higher score indicates the patients higher satisfaction.

#### 2.5.5. Comparison of No Results of Medical Staff before and after Intervention

Using our hospital's self-made questionnaire to evaluate the medical staff before and after the intervention with a five-point scale of 1–5 points, no results were obtained, including optimizing the dressing change process, team cohesion, work responsibility, and communication ability.

### 2.6. Statistical Processing

We used SPSS 22.0 software to process the data analysis of the patients included in this study, and the data on a linear scale were presented as mean ± standard deviation ($\bar{x}$ ±S). The two-sample independent *t*-test was used to compare the differences between groups without a time factor, and repeated measures were used. Analysis of variance was used to compare the differences between groups with time factor; enumeration data were expressed as rates, and differences between groups were compared by the *χ*^*2*^ test. *P* < 0.05 indicates a statistically significant difference.

## 3. Results

### 3.1. Comparison of Two Groups of General Data

There was no significant difference in age, sex, and surgical type between the two groups, as given in Table 1.

### 3.2. Comparison of Wound Repair Levels between the Two Groups of Patients

There was no significant difference in the wound area, wound depth, and VAS score between the groups combined with/without the medical-nursing integrated multidisciplinary-assisted surgical wound care model before surgery (*P* > 0.05). After 2 weeks of nursing and 4 weeks after nursing, the wound area, wound depth, and VAS score of the groups combined with/without the medical-nursing integrated multidisciplinary-assisted surgical wound care model continued to decrease and the group combined with the medical-nursing integrated multidisciplinary-assisted surgical wound care model lower than the group combined without the medical-nursing integrated multidisciplinary assisted surgical wound care model (*P* < 0.05), as shown in Figure 1.

### 3.3. Comparison of Wound Healing between the Two Groups of Patients

The granulation growth time, dressing change times, and wound healing time in the group combined with the medical-nursing integrated multidisciplinary-assisted surgical wound care model were all lower than those in the control group (*P* < 0.05), as shown in Figure 2.

### 3.4. Comparison of the Incidence of Complications between the Two Groups of Patients

The total complication rate of wound exudate, wound bleeding, nerve injury, and joint stiffness in the group combined with the medical-nursing integrated multidisciplinary-assisted surgical wound care model was 0.96%, which was significantly lower than that in the control group (6.25%) (*P* < 0.05), as shown in Figure 3.

### 3.5. Comparison of Patient Satisfaction Evaluation between Two Groups

The scores of hospitalization environment, medical and nursing professional level, work attitude, and psychological nursing satisfaction in the group combined with the medical-nursing integrated multidisciplinary-assisted surgical wound care model were higher than those in the control group (*P* < 0.05), as shown in Figure 4.

### 3.6. Comparison of No Results of Medical Staff before and after Intervention

After the intervention, the medical staff in optimizing the dressing change process, team cohesion, work responsibility, and communication ability were higher than those before the intervention (*P* < 0.05), as shown in Figure 5.

## 4. Discussion

Trauma refers to the tissue structure and damage caused by external factors acting on the body. In recent years, with the development of industry and economy in China, the turnover rate of surgical trauma beds increases year by year, which brings serious economic losses and disease burden to society and families [9, 10]. With the continuous development of medicine and nursing, attention has gradually been paid to the management of wound quality. At the same time, wound care of trauma patients after surgery has become the focus of clinical attention.

The medical care integrated multidisciplinary-assisted surgical wound care model is a combination of medicine, nursing, and nutrition and other multidisciplinary models to implement a full range of interventions for patients' surgical wound care, aiming to promote early recovery of patients [11, 12]. In the results of this study, after 2 weeks of nursing and 4 weeks of nursing, the wound area, wound depth, and VAS score of the two groups of patients were continuously decreased, and the observation group was lower than the control group (*P* < 0.05). It is suggested that the integration of medical care and multidisciplinary assistance in surgical wound care can promote the early healing of wounds and improve the pain level of patients. Previous studies have found that traumatic wounds are often accompanied by tissue fragments, dirt, and necrotic tissue, which aggravate the inflammatory response, cause severe pain in the body, and delay wound repair [13, 14]. In this study, a wound care team was quickly established after the patient was admitted to the hospital, and professionals from different disciplines such as attending physicians, nutritionists, rehabilitation specialists, and nurses were trained to learn wound types, healing, and evaluation. Observation, exercise, and dressing promote early wound healing. On the other hand, by establishing the optimal strategy for wound treatment and carrying out patient-centered support and treatment after injury recognition, postoperative wound infection was effectively controlled. Debridement and wound cleaning are practical techniques for controlling wound infection and can effectively reduce bacterial density. The traditional wound treatment mode is mostly operated by clinicians with less seniority, and its focus is on the cure of the disease while ignoring the subjective pain experience of patients. Nursing staff have more contact with patients in their daily work and have more obvious advantages in communication. They can dynamically assess patients' injuries by combining the relevant concepts of humanistic care and provide personalized nursing services; this also effectively relieves the pain [15].

Our study found that the time of granulation growth, the number of dressing changes, and the wound healing time in the observation group were lower than those in the control group, which suggests that the application of the nursing mode in the observation group would help the growth of new tissues and accelerate wound healing. Additionally, this study found that the total complication rate of wound exudate, wound bleeding, nerve injury, and joint stiffness in the observation group was 0.96%, which was significantly lower than that in the control group, which was 6.25%. Studies have shown that good cooperation between doctors and nurses can improve the quality of care, improve patient satisfaction, and improve patient clinical outcomes [16, 17]. In this study, the integrated medical care and multidisciplinary-assisted surgical wound care model have the following advantages. First, the application of appropriate wet wound dressings improved the wounding quality of debridement and dressing changes and reduced the overall complications of wound exudation, wound bleeding, nerve damage, and joint stiffness [18]. The incidence was significantly reduced, with good safety. The second one enhances the work enthusiasm of nurses, broadens their theoretical and operational knowledge, promotes the level of friendly cooperation between teams, and improves the cohesion between teams [19]. Combined with the results of this study, it can be shown that medical staff is optimizing the dressing change process after the intervention, team cohesion, work responsibility, and communication skills were higher than those before intervention. The third one improved the patient's level of satisfaction with nursing work. The results of this study showed that the observation group's scores on hospitalization environment, medical and nursing professional level, work attitude, and psychological nursing satisfaction were higher than those of the control group (*P* < 0.05). Traditional nursing work lacks effective communication, and most of the nursing staff execute the doctor's orders mechanically, which is easy to cause conflicts between doctors and patients and between nurses and patients [20]. In this study, the TCM physicians made medical orders after feedback from nurses after rounds, so that nurses could more accurately and effectively implement medical orders. In the process of discussion and analysis, nurses' understanding of patients' diseases could also be improved, and nursing care was improved. The quality of service has been recognized and praised by patients.

In conclusion, the medical-nursing integrated multidisciplinary-assisted surgical wound care model can improve the quality of patients' wound treatment and improve the patient's pain level, which is conducive to improving the cohesion of the medical and nursing team and the evaluation of patient's satisfaction. In addition, the shortcoming of this study lay in the short follow-up time, which could be extended in the future to further verify the results of this study.

## Figures and Tables

**Figure 1:** Comparison of wound area, wound depth, and VAS score between the two groups of patients after nursing (Note: ① Comparison of wound area between the two groups. ② Comparison of wound depth between the two groups. ③ Comparison of VAS scores between the two groups. Compared with the control group, ^*∗*^*P* < 0.05).

**Figure 2:** Comparison of wound healing between the two groups of patients (Note: compared with the control group, ^*∗*^*P* < 0.05).

**Figure 3:** Comparison of the incidence of complications between the two groups of patients.

**Figure 4:** Comparison of patient satisfaction scores between the two groups (Note: compared with the control group, ^*∗*^*P* < 0.05).

**Figure 5:** Comparison of no results of medical staff before and after intervention (Note: compared with before intervention, ^*∗*^*P* < 0.05).

**Table 1:** Comparison of two groups of general data.

Group	Gender (*n*)		Age (years)	Types of operations		
	Male	Female		Joint surgery	Spine surgery	Hand and foot surgery
Observation group (*n* = 96)	70	34	40.45 ± 4.22	29	35	40
Control group (*n* = 104)	63	33	40.36 ± 4.37	30	34	32
*χ* ^*2*^/*t*	0.063		0.148	0.601		
*P*	0.801		0.883	0.740		

## Data Availability

The data used to support the findings of this study are available from the corresponding author upon request.
